RETRACTED

# Evaluation of Anti-Obesity Activity, Acute Toxicity, and Subacute Toxicity of Probiotic Dark Tea

**DOI:** 10.3390/biom8040099

**Published:** 2018-09-25

**Authors:** Wang Ling, Shungeng Li, Xingcai Zhang, Yongquan Xu, Ying Gao, Qizhen Du, Guangguang Wang, Wentong Fan, Kai Sun, Jianchun Bian

**Affiliations:** 1 College of Veterinary Medicine, Yangzhou University, Yangzhou 225009, China; wl7590@163.com (W.L.); 18252736351@163.com (G.W.); fwtvetsz@sina.com (W.F.); m15705274808@163.com (K.S.); 2 Tianmu Lake Longxin Agricultural Ecological Park in Liyang City of Jiangsu Province, Liyang 213334, China; lishungengcool@163.com; 3 Jiangsu Co-innovation Canter for Prevention and Control of Important Animal Infectious Diseases and Zoonosis, Yangzhou 225009, China; 4 John A. Paulson School of Engineering and Applied Sciences, Harvard University, Cambridge, MA 02138, USA; 5 Tea Research Institute, Chinese Academy of Agricultural Sciences, 9 South Meiling Road, Hangzhou 310008, China; 6 College of Agricultural and Food Sciences, Zhejiang A & F University, Linan 311300, China

**Keywords:** probiotic dark tea, Sprague-Dawley (SD) rats, acute toxicity, subacute toxicity, anti-obesity, dyslipidemia

## Abstract

Probiotic dark tea (PDT) is a novel kind of dark tea produced by fresh albino tea leaves and fermented with specific probiotics. Our study demonstrates that PDT can ameliorate high-fat diet-induced overweight and lipid metabolic disorders and shows no acute or subacute toxicity in Sprague-Dawley (SD) rats. Daily intragastric administration of 5% PDT infusion for 14 days caused no obvious effect on general physiological features and behaviors of rats. Oral administration of 1%, 2%, and 3% of PDT infusion for six weeks had no influence on the biochemistry and histopathology of rats’ organs and blood, as well as the body weight and ratios of organ/body weight. To investigate its anti-obesity activity, SD rats were randomly divided into four groups, treated with normal diet + water (Group I), high-fat diet + water (Group II), high-fat diet + 3% traditional dark tea infusion (Group III), high-fat diet + 3% PDT infusion (Group IV). After six weeks, the body weight, serum total triacylglycerol (TG) and serum total cholesterol (TC) levels of rats in Group II were significantly increased and the high-density lipoprotein cholesterol (HDL) levels were significantly decreased compared with those in the other three groups. Both traditional dark tea and PDT treatment effectively counteracted the adverse effect of a high-fat diet in SD rats. These results suggest that PDT could be applied for the prevention of obesity, which ameliorates overweight and lipid metabolic disorders and which shows no acute or subacute toxicity.

RETRACTED

## 1. Introduction

Obesity is a medical condition in which excess body fat has accumulated to the extent that it may have a negative effect on health. The prevalence of obesity has doubled in more than 70 countries and has continuously increased in most other countries in the past 40 years [1]. In 2015, the population of obese children and obese adults were 107.7 million and 603.7 million, respectively [1]. China has the highest numbers of obese children and obese adults. Epidemiologic studies have demonstrated that obesity is a risk factor for many chronic diseases, such as cardiovascular, cancer, and musculoskeletal diseases [1]. Tea has been shown to be preventive to these diseases [2,3,4].

Dark tea is a class of tea that has undergone pile fermentation. During pile fermentation, the tea leaves are exposed to microbes in a high-humidity environment. Many components in tea leaves are degraded, oxidized, transformed and/or polymerized [5,6,7]. The alteration of these compounds affects the smell, taste, color and health-benefits of tea [8]. It is reported that some microbial metabolites in dark tea may ameliorate hyperlipidemia [9,10,11]. Some microbes may secrete enzymes (e.g., amylase, cellulose, pectase) to help produce water-soluble polysaccharides [12], which are capable of anti-obesity effects and modifying gut microbiota [13,14]. For example, during the pile fermentation, *Aspergillus niger* secrete massive cellulose and pectase, which effectively degrade polysaccharides, leading to increased contents of water-soluble polysaccharides in dark tea [15]. However, the safety of dark tea has become a major concern as microbes which can produce toxins are found during pile fermentation [3]. To solve this problem, probiotics with known ingredients, instead of microbes with unknown species, are added for the pile fermentation. Probiotic dark tea is a novel dark tea which is made of fresh albino tea leaves and fermented with specific probiotics *Eurotium cristatum*. The infusion of probiotic dark tea has mellow flavor, golden color and mellow taste. Compared with traditional dark tea, probiotic dark tea contains a higher content of prebiotics (e.g., polysaccharides).

In this study, the acute toxicity and subacute toxicity of probiotic dark tea was investigated to determine whether it could be regarded as a safe health-beneficial product. Later, the anti-obesity effect of probiotic dark tea was evaluated in high-fat diet Sprague-Dawley (SD) rat models. A comparison of the anti-obesity properties of probiotic dark tea and traditional dark tea was also made.

## 2. Materials and Methods

### 2.1. Materials

Traditional dark tea (first grade) was purchased from the tea market in Liyang, China. Probiotic dark tea was purchased from Longxing Ecological Agriculture Garden, Liyang, China. Normal diet pellets were purchased from Nanjing Anlimo Technology Co., Ltd. (Nanjing, China), while high-fat diet pellets (D12492, Rodent Diet with 60 kcal % Fat) were purchased from Shanghai Research Science Co., Ltd. (Shanghai, China). The total triglyceride assay kit, total cholesterol assay kit and high-density lipoprotein cholesterol assay kit were purchased from Nanjing Jiancheng Bioengineering Institute (Nanjing, China).

RETRACTED

Male Sprague-Dawley (SD) rats (four weeks old) weighing 80–100 g were purchased from the Experimental Animal Center of Jiangsu University (License No. SCXK (Su) 2013-0011, Yangzhou, China) and maintained at 22 ± 2 °C, 60 ± 10% humidity, natural light environment. The rats were fed with sterilized pellet diet and water *ad libitum*. The animals were acclimatized for two weeks under laboratory conditions. Ethical clearance for handling the animals was obtained from the ethical committee (Animal Care and Use Committee of Yangzhou University Approval ID: YDDW201606-002, Yangzhou, China) constituted for the purpose.

### 2.2. Methods

#### 2.2.1. Tea Infusion Preparation

Traditional dark tea or probiotic dark tea was mixed with distilled water at a designated proportion (i.e., 1%, 2%, 3% or 5%), incubated at 85 °C for 30 min. After filtration, the tea infusion was ready for further experiments.

#### 2.2.2. Acute Toxicity Studies

After two weeks of acclimation, 12 SD rats were randomly and evenly divided into two groups, treated with distilled water or 5% probiotic dark tea infusion at a dose of 5 mL/ (kg body weight × day) via intragastric administration for 14 days. The rats were monitored throughout the experiment, focusing on clinical appearances (e.g., behavior modification, skin lesions, feces) and death. An autopsy was carried out immediately after death. The food intakes of the rats were recorded every day and the body weight was measured every week. At the end of the observation period, the experimental rats were sacrificed after a 12 h fasting period and dissected for gross examination (including the organs’ size, color, consistency and other characteristics). Histological examination was undertaken if abnormal features were found.

#### 2.2.3. Subacute Toxicity Studies

The subacute oral toxicity studies were conducted according to GB 15670-1995. Briefly, after two weeks of acclimation, 24 SD rats were randomly and evenly divided into four groups, allowed free access to 1%, 2% or 3% probiotic dark tea or water, respectively, for six weeks. The body weight was measured every week. At the end of the experiment, animals were sacrificed after a 12 h fasting period. Blood samples were collected for complete blood counts, liver function tests and kidney function tests. The rats were then dissected for gross examination. The heart, liver, spleen, lung and kidneys of the rats were harvested and weighed to calculate relative organ weight (organ coefficients). 

RETRACTED

#### 2.2.4. The Anti-Obesity Effect of Probiotic Dark Tea in High-Fat Diet Sprague-Dawley Rats

After two weeks of acclimation, 24 SD rats were randomly and evenly divided into four groups, treated with normal diet + water (Group I), high-fat diet + water (Group II), high-fat diet + 3% dark tea infusion (Group III), high-fat diet + 3% probiotic dark tea infusion (Group IV) for six weeks. The food intakes and body weights were monitored every two days. At the end of the experiment, animals were sacrificed after a 12 h fasting period. Blood samples were collected to measure serum total triacylglycerol (TG), serum total cholesterol (TC) and high-density lipoprotein cholesterol (HDL) levels with corresponding kits, according to the manufacturer’s instructions, using an AU480 automatic biochemistry analyzer (Beckman Coulter, Brea, CA, USA).

#### 2.2.5. Statistical Analysis

All data were presented as means ± standard error of the mean (SEM) analyzed by one-way analysis of variance (ANOVA) followed by Dunnett’s test using SPSS 22.0 software (IBM, Chicago, IL, USA). *P* values less than 0.05 were considered significant.

## 3. Results

### 3.1. Acute Toxicity of Probiotic Dark Tea

The acute toxicity test showed no lethality or signs of toxicity for 5% probiotic dark tea. The food intake and body weight of rats were not affected by daily administration of 5% probiotic dark tea (Figure 1A,B). No abnormalities of organs in size, color, shape, consistency or other characteristics were observed through the gross examination. Thus, biochemical tests of blood and histopathological examinations of organs were not carried out. 

In a word, daily administration of probiotic dark tea at a dosage up to 5% was considered not acutely toxic. 

### 3.2. Subacute Toxicity of Probiotic Dark Tea

During the experiment, the behaviors, food intake, feces and hair of the rats to which probiotic dark tea was orally administered at a dosage up to 3% appeared normal. The body weight of rats which were administered probiotic dark tea was not different from that of rats in the control group, indicating oral administration of probiotic dark tea had no influence on the bioavailability of food (Figure 2A). 

At the end of the experiment, blood samples of rats were taken for various tests. An autopsy was carried out after the rats were sacrificed. Gross examination revealed that the shape, size and color of important organs (including heart, liver, spleen, lungs, kidneys, etc.) were normal, showing no signs of congestion, edema and necrosis. After morphological observation, the organs (including heart, liver, spleen, lungs and kidneys) were excised and weighed. The relative organ weights were all normal in rats which were administered probiotic dark tea (Figure 2B). This provides evidence that probiotic dark tea does not harm important organs in rats.

RETRACTED

The complete blood count tests revealed that, compared with the control group, no differences were found for the numbers of white blood cells (WBC), the numbers of lymphocytes (Lymph), the numbers of red blood cells (RBC), the content of hemoglobin (HGB), mean corpuscular volume (MCV), mean corpuscular hemoglobin concentration (MCHC), or the numbers of monocytes (Mon) in the rats administered probiotic dark tea at a dosage up to 3%. This shows that daily oral administration of up to 3% probiotic dark tea has no hematotoxicity in rats (Table 1). 

The results of liver function tests and kidney function tests showed no elevation of the levels of aspartate transaminase (AST), alkaline phosphatase (ALT), gamma glutamyl transpeptidase (GGT), total bilirubin (TBIL), blood urea nitrogen (BUN), total proteins (TP) and creatine kinase (CK) in the rats administered probiotic dark tea at a dosage up to 3% (Table 2). These data indicate that oral administration of up to 3% probiotic dark tea caused no hepatotoxicity or nephrotoxicity in rats.

In conclusion, oral administration of probiotic dark tea at a dosage up to 3% was not subacutely toxic. Therefore, 3% was the dose selected for evaluating the anti-obesity activity of probiotic dark tea in SD rats.

### 3.3. The Anti-Obesity Effect of Probiotic Dark Tea in High-Fat Diet Sprague-Dawley Rats

Both traditional dark tea and probiotic dark tea were observed to prevent high-fat diet-induced obesity. The average body weight of rats in Group II was much heavier than that in Group I (*p* < 0.05), indicating that a high-fat diet could induce overweight (Figure 3A). Compared with Group II, the average body weights of rats in Groups III and IV were significantly lighter. In fact, there was no significant difference among the average body weights of rats in Groups I, III and IV. No obvious difference was found between the average body weights of rats in Groups III and IV. This suggests that traditional dark tea and probiotic dark tea could effectively prevent the increase of body weight caused by a high-fat diet.

The serum total triacylglycerol and cholesterol levels of rats in Group II were significantly elevated (Figure 3B,C). Meanwhile, the HDL levels were notably lowered (Figure 3D). Oral administration of traditional dark tea or probiotic dark tea mitigated the increase of TG and TC, and the decrease of HDL (Figure 3B–D). Compared with traditional dark tea, probiotic dark tea showed stronger lipid-lowering activity.

RETRACTED

## 4. Discussion

Nowadays, people are paying more and more attention to food safety. The safety of traditional dark tea is doubtful as fungi that can produce carcinogens (e.g., ochratoxin A) are detected [16]. To solve this problem, modifications of the pile fermentation process are made to prevent toxic contamination. Instead of having a mixture of unknown bacteria and fungi, specific probiotics are added to tea leaves at the initiating stage of the pile fermentation. Probiotic dark tea is a kind of dark tea produced with modified pile fermentation. It contains not only the characteristics of dark tea but also the characteristics of prebiotics.

As a novel dark tea, its safety needed assessment. Acute toxicity and subacute toxicity tests were carried out in SD rats to evaluate the risk of short-term and long-term administration of probiotic dark tea, respectively. Daily intragastric administration of 5 mL/ (kg body weight), 5% probiotic dark tea for 14 days in rats, which was equal to daily oral administration of 0.083 g/ (kg body weight), 5% probiotic dark tea in humans, showed no distinct toxicity. No detectable body weight reduction, toxicity symptoms or death occurred. No obvious abnormality was found by gross examination of organs.

In the subacute toxicity study, rats were given free access to drink probiotic dark tea for six weeks. The body weight increase was not influenced by oral administration. No distinct abnormality in rats administered probiotic dark tea was observed by biochemical tests of blood samples (including complete blood count tests, liver function tests and kidney function tests) and histopathological examination of important organs. These results indicated that probiotic dark tea did not hamper the growth and development of rats, and did not cause hematotoxicity, hepatotoxicity or nephrotoxicity at the test doses. Relative organ weight analysis is an important endpoint for identification of potentially harmful effects of test compounds in toxicology studies [17]. In this study, the relative weights of key organs (e.g., heart, liver, spleen, lungs, kidneys) in rats administered probiotic dark tea were normal.

The above results demonstrated that probiotic dark tea had no acute toxicity or subacute toxicity at test doses. It can be regarded as a safe food and has the potential to be utilized in health-beneficial products.

RETRACTED

In previous studies, oral administration of 2–2.5% tea infusion could inhibit body weight increase, but had little effect on the regulation of blood lipids [18]. However, administration of tea infusion at higher dose could significantly reduce body weight and blood lipids without obvious toxicity [19,20]. In this study, the anti-obesity and lipid-lowering effect of 3% traditional dark tea and 3% probiotic dark tea were determined. Our results demonstrated that both traditional dark tea and probiotic dark tea reduced the body weight increase, serum total TG levels and serum total TC levels in high-fat diet SD rats. Compared with traditional dark tea, probiotic dark tea exhibited stronger activity in preventing the increase of serum total TC levels and elevating HDL levels. A former study revealed that intragastric administration of *E. cristatum* fermented Dark Tea Extract effectively decreased body weight and serum TG in the high-fat diet-induced rat model by targeting the peroxisome proliferators-activated receptors (PPAR) signaling pathway [21]. Our current study together with Liu’s study confirmed the weight-controlling effect of fermented dark tea and indicated that dark tea fermented with different species of microbes exerts its anti-obesity activity in different ways. *E. cristatum* fermented dark tea used in Liu’s study mainly regulated the serum TG levels, while probiotic dark tea used in this study not only reduced the serum TG levels, but also modulated the serum TC and high-density lipoprotein (HDL) levels. One of the predominant causes might be that different microbes produced and secreted different metabolites and enzymes.

Cholesterol is one of the major classes of lipids which all animal cells use to construct membranes [22]. All animal cells can manufacture cholesterol. Since cholesterol is water-insoluble, it is transported in the blood within lipoproteins [23,24]. There are several types of lipoproteins, including very low-density lipoproteins (VLDL), low density lipoproteins (LDL), intermediate density lipoproteins (IDL) and HDL. All of them can carry cholesterol. Increased levels of lipoproteins (except HDL) are associated with an increased risk of atherosclerosis and coronary heart disease [25]. However, elevated levels of HDL are associated with a reduced risk of cardiovascular diseases because HDL particles remove fat molecules from cells which need to export fat molecules, and transport it back to the liver for excretion or re-utilization [26,27]. Our study suggests that probiotic dark tea might prevent high-fat diet-induced hypercholesterolemia accelerating the removal of cholesterol in the blood through up-regulation of HDL.

RETRACTED

Nevertheless, which components play a central role in the anti-obesity and anti- hypercholesterolemia activity of probiotic dark tea remains unclear. The biomolecules related to the anti-obesity activity, acute toxicity, and subacute toxicity of probiotic dark tea can be attributed to polyphenols, polysaccharides, caffeine, etc. According to our knowledge, various components in dark tea, such as tea polyphenols, caffeine, theabrownins and polysaccharides, have been shown to reduce body weight increase and/or regulate blood lipids [28,29,30,31,32]. Previous studies show that polyphenols, polysaccharides, and caffeine can inhibit fatty acids absorption, reduce serum leptin levels, inhibit the interleukin-6 (IL-6) and tumor necrosis factor-alpha (TNF-α) gene expression, showing good anti-obesity property [32]. The above result is based on the study of green teas. In probiotic dark tea, the anti-obesity effect is more obvious, while the composition is much more complex than green tea. Compared with green tea, polyphenols, polysaccharides, and caffeine are still available in probiotic dark tea and are in a more highly condensed and concentrated form (e.g., theabrownins, theaflavin, thearubigins in probiotic dark tea as compared to catechins in green tea [2], which corresponds to its improved anti-obesity effect. More in-depth studies can be performed in this complex and important area to determine the most effective component(s) in the probiotic dark tea and explore the underlying mechanisms.

## 5. Conclusions

We produced a novel probiotic dark tea from fresh albino tea leaves with a specific probiotics fermentation process. Our results suggest that the probiotic tea can effectively counteract the adverse effect of high-fat diet in SD rats, thus ameliorating high-fat diet-induced overweight and lipid metabolic disorders. After six weeks, the body weight, serum total TG levels and serum TC levels of rats in the probiotic dark tea administered group were significantly increased and the HDL levels were significantly decreased compared with those in the other three groups. The probiotic tea showed no acute or subacute toxicity in SD rats. These results pave the way for new tea production and toxicity studies.

## Figures and Tables

**Figure 1:** Effect of daily administration of 5% probiotic dark tea for 14 days on the food intake (**A**) and body weight (**B**) of Sprague-Dawley (SD) rats.

**Figure 2:** Effect of daily administration of 1%, 2% and 3% probiotic dark tea for six weeks on the body weight (**A**) and relative organ weights (**B**) of SD rats.

**Figure 3:** Effect of traditional dark tea and probiotic dark tea on the body weight (**A**), serum total cholesterol levels (**B**), serum total triglyceride levels (**C**) and serum high density lipoprotein cholesterol levels (**D**) of high-fat diet SD rats. *, ** represents statistical significance at *p* < 0.05, *p* < 0.01, compared with Group Ι, respectively; #, ## represents statistical significance at *p* < 0.05, *p* < 0.01, compared with Group II, respectively.

RETRACTED

**Table 1:** Results of complete blood counts of Sprague-Dawley (SD) rats administered probiotic dark tea (PDT).

Group	WBC (10^9^/L)	Lymph (%)	RBC (10^12^/L)	HGB (g/L)	MCV (Fl)	MCHC (g/L)	Mon (%)
Control	4.67 ± 0.78	75.38 ± 3.16	6.97 ± 0.65	140.00 ± 7.59	55.22 ± 1.50	307.33 ± 5.32	2.82 ± 0.29
1% PDT	4.70 ± 1.04	75.80 ± 6.59	7.12 ± 0.65	134.33 ± 12.13	55.92 ± 0.70	316.33 ± 7.74	3.05 ± 0.73
2% PDT	4.45 ± 1.45	75.47 ± 4.53	7.19 ± 0.28	138.33 ± 9.91	54.75 ± 1.71	320.50 ± 12.94	3.23 ± 0.93
3% PDT	4.97 ± 1.01	74.73 ± 4.84	6.93 ± 0.96	136.67 ± 5.13	56.17 ± 1.61	309.67 ± 7.06	2.67 ± 0.66

Notes to abbreviations: white blood cells (WBC), the numbers of lymphocytes (Lymph), the numbers of red blood cells (RBC), the content of hemoglobin (HGB), mean corpuscular volume (MCV), mean corpuscular hemoglobin concentration (MCHC), the numbers of monocytes (Mon).

**Table 2:** Results of liver function tests and kidney function tests of SD rats administered PDT.

Group	ALT (U/L)	AST (U/L)	GGT (U/L)	TBIL (μmol/L)	TP (g/L)	CK (U/L)	BUN (mmol/L)
Control	64.76 ± 14.77	42.98 ± 3.30	5.00 ± 0.71	4.54 ± 1.21	80.52 ± 2.08	160.40 ± 26.69	4.87 ± 0.57
1%PDT	53.12 ± 16.34	36.80 ± 4.25	3.12 ± 2.07	6.60 ± 3.83	76.55 ± 3.07	138.17 ± 26.07	5.89 ± 0.82
2%PDT	52.50 ± 15.27	40.32 ± 7.53	3.77 ± 1.30	4.77 ± 1.93	76.23 ± 3.77	128.83 ± 22.56	5.78 ± 0.73
3%PDT	71.68 ± 16.29	38.18 ± 5.31	4.22 ± 1.65	6.67 ± 1.67	77.55 ± 4.08	167.67 ± 33.13	5.59 ± 1.96

Notes to abbreviations: alkaline phosphatase (ALT), aspartate transaminase (AST), gamma glutamyl transpeptidase (GGT), total bilirubin (TBIL), total proteins (TP), creatine kinase (CK), and blood urea nitrogen (BUN).
